The article "Systematic Evaluation Meta-Analysis of the Efficacy of Recombinant Human Endostatin Combined with Gemcitabine and Cisplatin in Non-Small-Cell Lung Cancer" was published in 2022. Journal: J Healthc Eng.

# Systematic Evaluation Meta-Analysis of the Efficacy of Recombinant Human Endostatin Combined with Gemcitabine and Cisplatin in Non-Small-Cell Lung Cancer

**DOI:** 10.1155/2022/3208780

**Published:** 2022-03-15

**Authors:** Li Zhang, Yuan He, ChengFeng Yi, Mei Huang

**Affiliations:** Yunyang County People's Hospital Oncology Department, Chongqing, China

## Abstract

**Objective:**

To evaluate the efficacy of recombinant human endostatin combined with gemcitabine and cisplatin in the treatment of non-small-cell lung cancer (NSCLC).

**Methods:**

The databases of Cochrane Library, Embase, ClinicalTrials, PubMed, HowNet, Wanfang, and VIP were searched to collect randomized controlled trials (RCTs) of recombinant human endostatin combined with gemcitabine and cisplatin (experimental group) and gemcitabine combined with cisplatin (control group) for comparative study. The quality of literature was evaluated by bias risk assessment tools and related scales, and then meta-analysis was performed.

**Results:**

A total of 27 RCTs (1646 patients) were included. The results of meta-analysis showed that the effective rate (*P* < 0.000 01) and benefit rate (*P* < 0.000 01) of the experimental group were significantly higher than those of the control group, the incidence of leucopenia (*P* = 0.79), thrombocytopenia (*P* = 0.39), and gastrointestinal reaction (*P* = 0.85) were not statistically significant.

**Conclusion:**

The combination of recombinant human endostatin, gemcitabine, and cisplatin can increase the efficacy and safety of NSCLC patients.

## 1. Introduction

Nowadays, the prevalence trend and death status of lung cancer are not optimistic. Non-small-cell lung cancer (NSCLC) accounts for about 4/5 of all lung cancer patients, which is a cancer with high mortality in the world. The first-line chemotherapy of NSCLC is vinorelbine, gemcitabine, and cisplatin, which is widely used [1]. However, chemotherapy drugs are generally cytotoxic. Although they have a destructive effect on lung cancer cells, they also limit human immunity. In the process of lung cancer chemotherapy, it is a difficult problem for NSCLC to ensure the curative effect and reduce the adverse reactions as much as possible. Chemotherapy is the main treatment for advanced NSCLC patients. The standard treatment is 4–6 cycles of platinum combined with the third generation of cytotoxic drugs. The effective rate is 20.00%–30.00% [2]. The median survival time is 8–10 months, and the time of disease progression is 3–5 months. To some extent, the survival time of NSCLC patients can be prolonged, but the curative effect has reached the plateau [3, 4]. Therefore, in order to improve the survival and efficiency of patients with advanced NSCLC, we need to try new drugs and new chemotherapy regimens that are different from the existing treatment mechanisms. It is against this background that antitumor angiogenesis therapy is produced. Since the role of angiogenesis in tumor growth and progression was identified in the 1970s, the exploration of antiangiogenic drugs has not been interrupted [5]. With the progress of science and technology, many antiangiogenic drugs have been developed and applied in clinic. A large number of clinical studies have confirmed that the combination of molecular targeted drugs and chemotherapy can achieve the above therapeutic purposes, and some reports have shown that these drugs have a certain effect on tumor vascular normalization and can increase the sensitivity to chemotherapy and radiotherapy; when combined with chemotherapy, it has a positive synergistic effect. Recombinant human endostatin, also known as endostatin, is an angiogenesis inhibitor, which can inhibit angiogenesis and limit tumor angiogenesis. Nowadays, recombinant human endostatin can be used to intervene in NSCLC, gastric cancer, and so on [6]. Studies have shown that recombinant human endostatin and chemotherapy drugs can play a synergistic effect, making the efficacy increase. Although targeted therapy combined with chemotherapy has achieved a positive therapeutic effect in clinic, antiangiogenesis therapy has not achieved the obvious antitumor effect as in the animal experiment stage. There are many factors related to its possibility, but the difference in drug use is one of the most important factors [7]. Conventional drugs are treated by intravenous route. After the combination of drugs with plasma protein, the concentration of drugs distributed to the local tumor is significantly reduced, and the therapeutic effect of the tumor is not good. Interventional targeted therapy of tumor blood supply artery is a mature method of local perfusion chemotherapy [8]. This method is through superselective intubation to the target artery of tumor blood supply, a high concentration of therapeutic drugs is infused into the tumor area. Through the first-pass effect of drugs, the concentration of drugs in the tumor is increased; the action time is prolonged; the clinical side effects are reduced; and the tolerance of patients is increased. It is believed that endostatin combined with chemotherapeutic drugs can significantly increase the clinical therapeutic effect of NSCLC. In this study, we systematically reviewed the efficacy of recombinant human endostatin, gemcitabine, and cisplatin combined therapy and gemcitabine and cisplatin combined therapy in the treatment of NSCLC.

The article "Systematic Evaluation Meta-Analysis of the Efficacy of Recombinant Human Endostatin Combined with Gemcitabine and Cisplatin in Non-Small-Cell Lung Cancer" was published in 2022. Journal: J Healthc Eng.

## 2. Information and Methods

### 2.1. Inclusion Criteria and Exclusion Criteria

#### 2.1.1. Inclusion Criteria

The inclusion criteria are as follows: (1) randomized controlled trials (RCTs) were published in Chinese and English; (2) cytological or histopathological diagnosis of NSCLC was made, regardless of gender, age, course of disease, and so on; (3) the blood routine, heart, liver, kidney, and brain function were basically normal, and there were no structural or functional abnormalities of important organs; and (4) the period of treatment is no less than 2 cycles (1 cycle is 2 weeks).

#### 2.1.2. Exclusion Criteria

The exclusion criteria are as follows: (1) the score of the Jadad scale was 0 or non-RCT literature, (2) repetitive literature, (3) descriptive research, (4) impossible to extract literature, and (5) animal experiments.

#### 2.1.3. Method

The control group was treated with gemcitabine and cisplatin; patients in the experimental group were treated with gemcitabine, cisplatin, and recombinant human endostatin.

#### 2.1.4. Outcome Measures

(1) Total effective rate, (2) benefit rate, (3) the incidence of leukopenia, (4) the incidence of thrombocytopenia, and (5) the incidence of gastrointestinal reactions are calculated. According to the new criteria for evaluation of solid tumor efficacy, the efficacy criteria were divided into complete remission (CR), partial remission (PR), steady (SD), and advanced (PD). Effective rate = (Cr + PR)/total cases × 100.00%; benefit rate = (Cr + PR + SD)/total cases × 100.00%; the incidence of leukopenia = 1–4 cases/total cases × 100.00%; and incidence of thrombocytopenia = cases of grade 1–4/total cases × 100.00%.

### 2.2. Literature Retrieval

A total of 501 databases of Cochrane Library, Embase, ClinicalTrials, PubMed, HowNet, Wanfang, and VIP are searched. Of these, 404 were included, and 97 were excluded. The Chinese keywords are “recombinant human angiostatin,” “non-small cell lung cancer,” “gemcitabine,” “cisplatin,” “meta-analysis,” and so on. The English keywords are “recombinant human endostatin,” “non-small cell lung cancer,” “gemcitabine,” “cisplatin,” and “meta-analysis.” The retrieval time period is from the establishment of each database to October 2020.

### 2.3. Screening of the Literature and Data

A total of three reviewers screened and checked the literature; two of them independently screened the literature according to the inclusion criteria and exclusion criteria; and two of them checked the literature. The third reviewer assisted in the case of different opinions. The extracted information included the year of publication, first author, sample size, age range, intervention method, disease stage, intervention course, outcome index, and so on.

The article "Systematic Evaluation Meta-Analysis of the Efficacy of Recombinant Human Endostatin Combined with Gemcitabine and Cisplatin in Non-Small-Cell Lung Cancer" was published in 2022. Journal: J Healthc Eng.

### 2.4. Literature Quality Assessment

The Cochrane system version 5.1.0 was used to assess the risk of bias, whether the distribution was hidden, whether blinding was used (blinding of investigators and subjects and blinded assessment of the final results of the study), whether the results from the data were complete, whether the results of the study were selectively reported, and whether there were other sources of bias. Each item has a low risk of bias, ambiguity, and high risk of bias. Jadad scale was used to evaluate the quality of the study, including random sequence generation (appropriate 2 points, uncertain 1 points, and inappropriate 0 points), randomized concealment (appropriate 2 points, uncertain 1 points, and inappropriate 0 points), blind method (appropriate 2 points, uncertain 1 points, and inappropriate 0 points), withdrawal and withdrawal (description 1 points, no description, and 0 points). The score of low-quality research is less than 3, and that of high-quality research is 4–7.

### 2.5. Statistical Methods

Revman 5.3 software was used to analyze the data. The relative risk (RR) or odds ratio (or) and 95% confidence interval (CI) were used as the combined effect quantity if the included indexes were binary variables; if the included research indicators were continuous variables, they were expressed by weight mean difference (MD) or standard mean difference (SMD) and 95% CI. For the heterogeneity analysis of the included studies, when the heterogeneity among the studies was low (*I*^2^ ≤ 50%), the fixed-effect model was used for meta-analysis; when the heterogeneity among the studies was relatively high (*I*^2^ > 50%), the random-effects model was used for meta-analysis, and the incomplete data were used for descriptive analysis. The bias was analyzed qualitatively by funnel plot and quantitatively by state 12.0.

## 3. Results

### 3.1. Results of Literature Search

A total of 360 literature were collected, including 317 in Chinese and 43 in English. After reading the title and abstract, 81 related articles were obtained. After careful study of the full text, 27 articles were finally included, including 1,646 subjects, 830 patients in the experimental group, and 816 patients in the control group (Figure 1). The basic information of the study is shown in Table 1.

### 3.2. Assessment of the Quality of Included Studies

All studies were RCTs; among them, six studies involved randomized methods, and none of them involved allocation concealment, blind method, or other sources of bias. See Figures 2 and 3 for details.

### 3.3. Results of Meta-Analysis

#### 3.3.1. Efficiency

Among them, 27 studies related to the effective rate, which had no statistical heterogeneity (*P* = 0.99, *I*^2^ = 0). The fixed-effect model was used for the meta-analysis, as shown in Table 2. The results of meta-analysis showed that the effective rate of the experimental group was significantly higher than that of the control group, with statistical significance (RR = 1.67, 95% CI (1.48, 1.89), *P* < 0.00001).

The article "Systematic Evaluation Meta-Analysis of the Efficacy of Recombinant Human Endostatin Combined with Gemcitabine and Cisplatin in Non-Small-Cell Lung Cancer" was published in 2022. Journal: J Healthc Eng.

#### 3.3.2. Clinical Benefit Rate

Among them, 27 studies related to the benefit rate, which had no statistical heterogeneity (*P* = 0.49, *I*^2^ = 0). The fixed-effect model was used for the meta-analysis, as shown in Table 3. The results of meta-analysis showed that the benefit rate of the experimental group was significantly higher than that of the control group (RR = 1.26, 95% CI (1.20, 1.33), *P* < 0.00001).

#### 3.3.3. Incidence of Leukopenia

Among them, 19 studies related to the incidence of leukopenia, which was not statistically heterogeneous (*P* = 1.00, *I*^2^ = 0). The fixed effect model was used for meta-analysis. Meta-analysis showed that the incidence of leukopenia among the groups was not statistically significant (RR = 0.98, 95% CI (0.88, 1.11), *P* = 0.79).

### 3.4. Bias Analysis

Take the effective rate as an index and use the inverted funnel plot and Begg's test to analyze the bias, as shown in Figures 4 and 5. It can be seen from Figure 5 that all the scattered points in the study are within the scope of the inverted funnel diagram, and the distribution is basically symmetrical, indicating that there is a small possibility of bias in this study. Figure 5 shows that the *P* value of Begg's test is 0.084 > 0.05, indicating that there is no obvious bias in this study.

## 4. Discussion

Lung cancer is the most malignant tumor in China and has the highest incidence rate in the world [9]. Most patients have an advanced tumor at the time of diagnosis, and NSCLC accounts for 80.00% of lung cancer in the late stage. Because the prognosis of NSCLC is not ideal, its treatment is very challenging [10]. Treatment of advanced NSCLC has also experienced a process. In 1980s, there were serious side effects of the first-generation chemotherapy drugs (cyclophosphamide, etc.); a clinical study showed that the prognosis after the first-generation chemotherapy drug treatment was not significantly improved compared with the patients with the best support treatment [11]. Therefore, it was generally considered that support therapy was the best treatment method for advanced NSCLC. The idea lasted until 1995; a meta-analysis published in the British Journal of medicine confirmed for the first time that platinum-containing chemotherapy significantly improved the survival time of patients with advanced NSCLC than the best support therapy [12]. This meta-analysis was selected into 52 randomized controlled studies, including 9,387 NSCLC patients. The results showed that the death risk and 1-year survival rate were improved by 10.00% (*P* < 0.0001) after chemotherapy with platinum in patients with advanced NSCLC. The results of the analysis of the effects of chemotherapy on the survival of 2,714 patients with advanced NSCLC in 16 randomized controlled studies showed that chemotherapy combined with support therapy reduced the risk of death by 23.00% (*P* < 0.0001); the total survival time was prolonged by 1.50 months, and the 1-year survival rate was improved by 9.00% [13]. The results fully show that chemotherapy based on platinum drugs can reduce the risk of death and bring obvious survival benefits to patients, thus promoting NSCLC treatment into platinum-containing chemotherapy era. Among the above chemotherapy schemes, gemcitabine + cisplatin (GP) has some advantages. In 2005, Le Chavalier et al. conducted a meta-analysis of a single study of gemcitabine plus platinum-based chemotherapy and other platinum-containing chemotherapy options to assess whether there is a treatment that is more advantageous in advanced NSCLC [14]. The meta-analysis was selected into 13 studies (4,500 cases), except for two phase II studies, all of which were phase III studies. Five studies were cisplatin single drug or first and second generation combined platinum-containing programs (1,900 cases), and 8 were third generation combined platinum (2,600 cases). The results showed that GP could significantly reduce the disease progression and death risk by 12.00% and 10.00%, respectively, compared with other chemotherapy schemes; compared with the first and second generation combined platinum-containing regimen, GP could significantly prolong the total survival period of patients (*P* < 0.001); and compared with other third-generation platinum-containing regimen without gemcitabine, gemcitabine significantly prolonged the progression-free survival period (*P* < 0.001). The results of this analysis fully confirm that gemcitabine plus platinum combined regimen can significantly prolong the total and progression-free survival of patients with advanced NSCLC compared with other platinum-containing schemes. In 2007, Grossi et al.'s meta-analysis compared the activity of gemcitabine with three other third-generation platinum-containing chemotherapy programs [15]. The meta-analysis included 48 studies, with 6,671 patients. The results showed that gemcitabine could significantly reduce the risk of disease progression by 14.00% compared with other third-generation platinum-containing chemotherapy. This meta-analysis study not only laid the foundation position of platinum-containing chemotherapy in advanced NSCLC treatment but also highlighted the treatment advantages of GP. Patients with advanced NSCLC received gemcitabine plus platinum first-line treatment, which can achieve a higher quality of life and longer life [16]. Therefore, GP with small side effects and good tolerance was used as chemotherapy. But there is no essential difference in efficacy between the third-generation chemotherapy drugs and platinum. The randomized controlled study ECoG 1594, published in the New England Journal of medicine in 2002, showed that there was no significant difference in the median OS between the four third-generation platinum-containing chemotherapy regimens (gemcitabine, paclitaxel, docetaxel, and vinorelbine combined with platinum) [17]. The treatment cycle of the first-line chemotherapy program and the combination of three chemotherapy drugs were also confirmed by the phase II clinical study of MPCRN cancer research network in the United States [18]. Therefore, if we want to further improve the chemotherapy effect of lung cancer, we must take new ideas.

The article "Systematic Evaluation Meta-Analysis of the Efficacy of Recombinant Human Endostatin Combined with Gemcitabine and Cisplatin in Non-Small-Cell Lung Cancer" was published in 2022. Journal: J Healthc Eng.

The growth and diffusion of cancer cells depend on angiogenesis and tumor neogenesis, which is the most important antitumor method of vascular targeted therapy [19, 20]. In some studies, NSCLC patients were divided into 34 cases of platinum chemotherapy and 54 cases of platinum plus recombinant human endostatin [21–23]. It was found that the progression-free survival rate and overall survival rate of patients treated with combination therapy were significantly improved. Other related studies have pointed out that the efficacy of combined therapy is controversial and needs further study [24]. Gemcitabine is a substitute for inhibitory enzymes, which can inhibit the DNA replication of tumor cells in the process of DNA synthesis and repair. In order to study the curative effect of recombinant human endostatin in patients with NSCLC, this study summarized the randomized controlled trials of chemotherapy regimens in patients with NSCLC. The results showed that recombinant human endostatin combined with gemcitabine and cisplatin could significantly improve the total effective rate and benefit rate, and the bias analysis of funnel plot and Egger's test showed that the results were more reliable. The incidence of leucopenia, thrombocytopenia, and gastrointestinal reactions between the two groups were not statistically significant, indicating that the combination of recombinant human endostatin, gemcitabine, and cisplatin is safe [25].

The article "Systematic Evaluation Meta-Analysis of the Efficacy of Recombinant Human Endostatin Combined with Gemcitabine and Cisplatin in Non-Small-Cell Lung Cancer" was published in 2022. Journal: J Healthc Eng.

Ouyang Lihui et al. conducted a meta-analysis in 2012 to compare the efficacy of gemcitabine + cisplatin + recombinant human endostatin (GPE) regimen and gemcitabine + cisplatin (GP) regimen in patients with NSCLC; GPE is superior to GP in total effective rate and disease control rate. Ma et al. included 9 studies and 839 patients with NSCLC [26]. The results showed that the GPE regimen did not increase the incidence of adverse reactions compared with the GP regimen. The combined results of 4 studies found that compared with the GP scheme, the GPE scheme led to increased arrhythmia, and the difference was statistically significant. This suggests that clinicians should pay close attention to the ECG of patients with NSCLC when using a GPE regimen to prevent serious adverse reactions of arrhythmia. At the same time, the log-rank test was used to compare the disease progression and overall survival of the two groups. It was found that recombinant human endostatin combined with GP regimen did not improve the overall survival of patients with advanced NSCLC, but it did not exclude the bias caused by the small sample size of this study, and it was also affected by the later treatment effect of patients. The main adverse reactions of recombinant human endostatin combined with GP regimen to patients with advanced NSCLC were myelosuppression and gastrointestinal reactions. A few patients had liver function damage and ECG changes, but there was no significant difference compared with patients treated with GP regimen alone.

The curative effect of recombinant human endostatin, gemcitabine, and cisplatin in the treatment of patients with NSCLC has been improved, without obvious adverse reactions. The disadvantages are as follows: firstly, the unpublished literature are not included; secondly, the comprehensive quality evaluation of the included literature is low; thirdly, the included literature are all Chinese literature, which are not suitable for foreign patients; and fourthly, the quality of life evaluation of patients is not involved.

## 5. Conclusion

The combination of recombinant human endostatin, gemcitabine, and cisplatin can increase the efficacy and safety of NSCLC patients.

## Figures and Tables

**Figure 1:** Flow chart.

**Figure 2:** Bar chart of bias risk.

**Figure 3:** Bias risk diagram.

**Figure 4:** Inverted funnel plot of effective rate.

**Figure 5:** Efficient Begg's diagram.

**Table 1:** Basic information of the study.

Year of publication and first author	Number of cases		Age (years)		Method		Intervention course (d)	Outcome measures	Jadad score (points)
	Control group	Experimental group	Control group	Experimental group	Control group	Experimental group			
Tan Yong in 2013	38	38	61.70 ± 9.80		Gemcitabine 1,000 mg, intravenous drip, once daily, *d*_1–8_ + cisplatin 25 mg/m^2^, intravenous drip, once daily, *D*_1–3_	The control group was treated with the chemotherapy regimen + recombinant human endostatin 7.50 mg/m^2^, 0.9% sodium chloride injection 500 ml, intravenous drip, once a day, *d*_1–14_	21	(1) (2) (3) (4) (5)	3
Xie Yanru in 2009	26	22	44.00–71.00	44.00–69.00	Gemcitabine 1,000 mg, *D*_1_, *D*_8_ + cisplatin 75 mg/m^2^, divided into three days	The control group was treated with the chemotherapy regimen + recombinant human endostatin 15 mg, 0.9% sodium chloride injection 500 ml, intravenous drip, *d*_1–14_	21	(1) (2) (3) (4) (5)	2
Chen Yongxing in 2010	25	30	49.00 ± 3.00	50.00 ± 2.00	Gemcitabine 1,000 mg, IV, *D*_1_, *D*_8_ + cisplatin 25 mg/m^2^, IV, *D*_1–3_	The control group was treated with the chemotherapy regimen + recombinant human endostatin 15 mg, added with 0.9% sodium chloride solution 500 ml, intravenous drip, *d*_1–14_	21	(1) (2) (3) (4) (5)	1
Gu Ying in 2010	33	27	53.60		Gemcitabine 1,000 mg/m^2^, *D*_1_, *D*_8_ + cisplatin 25 mg/m^2^, intravenous drip, *D*_1–3_	The control group was treated with the chemotherapy regimen + recombinant human endostatin 15 mg, added with 0.9% sodium chloride solution 500 ml, intravenous drip, *d*_1–14_	21	(1) (2) (3) (4) (5)	1
Guo Hongbin in 2010	38	38	55.00 ± 12.00	53.00 ± 14.00	Gemcitabine 1,000 mg/m^2^, intravenous drip, *D*_1_, *D*_8_ + cisplatin 30 mg/m^2^, intravenous drip, *D*_1–3_	The control group was treated with the chemotherapy regimen + recombinant human endostatin 15 mg, intravenous drip, *d*_1–14_	21	(1) (2) (3) (4)	2
Wei Qihong in 2010	16	16	59.80		Gemcitabine 1 g/m^2^, intravenous drip, *D*_1_, *D*_8_ + cisplatin 30 mg/m^2^, intravenous drip, *d*_2–4_	The control group was treated with the chemotherapy regimen + recombinant human endostatin 15 mg, intravenous drip, once a day, *d*_1–14_	21	(1) (2) (3) (4) (5)	2
Xu Jian in 2010	20	20	64.00		Gemcitabine 1,000 mg/*M*^2^ + cisplatin 30 mg/m^2^, tumor target artery perfusion, *D*_1_, gemcitabine 1,000 mg/m^2^, IV, *D*_8_, 0.9% sodium chloride injection 500 ml, intravenous drip, *D*_2–12_	The control group was treated with the chemotherapy regimen + recombinant human endostatin 15 mg/*D*, 0.9% sodium chloride injection 500 ml, intravenous drip, 2–12 days	36	(1) (2) (3) (4) (5)	2
Chen Qun in 2011	35	33	65	63	Gemcitabine 1,000 mg/m^2^, intravenous drip, *D*_1_, *D*_8_ + cisplatin 80 mg/m^2^, intravenous drip, *D*_1_	The control group was treated with the chemotherapy regimen + recombinant human endostatin 15 mg, 0.9% sodium chloride solution 500 ml, intravenous drip, *d*_1–14_, intermittent for 7 days	21	(1) (2) (3) (4) (5)	1
Ruan Mei in 2011	19	17	58.50		Gemcitabine 1,000 mg/m^2^, *D*_1_, *D*_8_ + cisplatin 75 mg/m^2^, divided into three days	The control group was treated with the chemotherapy regimen + recombinant human endostatin 15 mg, 0.9% sodium chloride injection 500 ml, intravenous drip, *d*_1–14_	21	(1) (2) (3) (4) (5)	1
Wang Fen in 2011	29	31	55.00	56.00	Gemcitabine 1,000 mg/m^2^, IV, *D*_1_, *D*_8_ + cisplatin 75 mg/m^2^, IV, *D*_1_	The control group was treated with the chemotherapy regimen + recombinant human endostatin 15 mg, 0.9% sodium chloride solution 500 ml, intravenous drip, *d*_1–14_, intermittent for 7 days	21	(1) (2)	1
Zheng Qingping in 2011	18	17	54.50	50.10	Gemcitabine 1,000 mg/m^2^, intravenous drip, *D*_1_, *D*_8_ + cisplatin 20 mg/m^2^, intravenous drip, *D*_1–5_	The control group was treated with the chemotherapy regimen + recombinant human endostatin 15 mg/*D*, intravenous drip, *d*_1–14_	21–28	(1) (2) (5)	1
Chen Bing in 2012	26	27	56.50 ± 7.30	55.70 ± 8.60	Gemcitabine 1,000 mg/m^2^, 0.9% sodium chloride injection 100 ml, intravenous drip, *D*_1_, *D*_8_ + cisplatin 25 mg/m^2^, 0.9% sodium chloride injection 500 ml, intravenous drip, *d*_2–4_	The control group was treated with the chemotherapy regimen + recombinant human endostatin 15 mg, intravenous drip, once a day, *d*_1–14_	14	(1) (2) (3) (4) (5)	1
He Rong in 2012	32	40	69.80 ± 5.50	70.50 ± 5.30	Gemcitabine 1,000 mg/m^2^, *D*_1_, *D*_8_ + cisplatin 30 mg/m^2^, *d*_2–4_	The control group was treated with the chemotherapy + recombinant human endostatin 7.50 mg/m^2^, *d*_1∼14_	21	(1) (2) (5)	1
Liu Jianwu in 2012	30	30	56.00	58.00	Gemcitabine 1,000 mg/m^2^, IV, *D*_1_, *D*_8_ + cisplatin 75 mg/m^2^, IV, *D*_1_, *D*_2_	The control group was treated with the chemotherapy + recombinant human endostatin 15 mg, *D*_1–7_	21	(1) (2) (3) (4) (5)	2
Luan Wenqiang in 2012	27	25	40.00–67.00	42.00–68.00	Gemcitabine 1,250 mg/m^2^, IV, *D*_1_, *D*_8_ + cisplatin 75 mg/m^2^, IV, *D*_1_	The control group was treated with the chemotherapy regimen + recombinant human endostatin 75 mg/m^2^, added with 0.9% sodium chloride solution 500 ml, intravenous drip, *d*_1–14_	21	(1) (2)	1
Yin Feng in 2012	90	94	49.30 ± 4.50	48.30 ± 5.20	Gemcitabine 1,000 mg/m^2^, intravenous drip, *D*_1_, *d*_8_ + cisplatin 30 mg/m^2^, intravenous drip, *d*_2–4_	The control group was treated with the chemotherapy regimen + recombinant human endostatin 15 mg, 0.9% sodium chloride injection 500 ml, intravenous drip, once a day, *d*_1–14_	21	(1) (2) (5)	1
Almu Jiang in 2013	40	40	59.20 ± 9.50	58.30 ± 9.60	Gemcitabine 1.00 mg/m^2^, 0.9% sodium chloride injection 250 ml, intravenous drip, *D*_1_, *D*_14_ + cisplatin, 0.9% sodium chloride injection 500 ml, intravenous drip, *D*_1–3_	The control group was treated with the chemotherapy regimen + recombinant human endostatin 15 mg, 0.9% sodium chloride injection 500 ml, intravenous drip, *d*_1–14_	21	(1) (2) (3) (4) (5)	2
Zhang Yuanyuan in 2014	28	31	54.00	53.00	Gemcitabine 1,000 mg/m^2^, *D*_1_, *D*_8_ + cisplatin 75 mg/m^2^, divided into three days	The control group was treated with the chemotherapy regimen + recombinant human endostatin 15 mg, 0.9% sodium chloride injection 250 ml, intravenously pumped, *d*_1–9_	21	(1) (2) (3) (4) (5)	2
Fu Hao in 2015	28	32	55.81	56.21	Gemcitabine 1,000 mg/m^2^, intravenous drip, *D*_1_, *D*_8_ + cisplatin 25 mg/m^2^, intravenous drip, *D*_1–3_	The control group was treated with the chemotherapy regimen + recombinant human endostatin 15 mg, 0.9% sodium chloride injection 500 ml, intravenous drip, *d*_1–14_, intermittent for 7 days	21	(1) (2) (3) (4) (5)	2
Liu Tao in 2015	32	32	No explanation		Gemcitabine 1,000 mg/m^2^, intravenous drip, *D*_1_, *D*_8_ + cisplatin 80 mg/m^2^, intravenous drip, *D*_1_, *D*_2_	The control group was treated with the chemotherapy regimen + recombinant human endostatin 15 mg, added with 0.9% sodium chloride injection 500 ml, *d*_1–14_, repeated intermittently for 7 days	21	(1) (2)	2
Li Lihua in 2016	23	23	52.30 ± 10.60		Gemcitabine 1,000 mg/m^2^, intravenous drip, *D*_1_, *D*_8_ + cisplatin 30 mg/m^2^, intravenous drip, *D*_1–3_	The control group was treated with the chemotherapy regimen + recombinant human endostatin 15 mg, 0.9% sodium chloride solution 500 ml, intravenous drip, *d*_1–14_, intermittent for 7 days	21	(1) (2) (3) (4) (5)	3
Fangli in 2017	23	23	52.00	60.00	Gemcitabine 1,000 mg/m^2^, intravenous drip, *D*_1_, *D*_8_ + cisplatin 75 mg/m^2^, intravenous drip, *D*_1–3_	The control group was treated with the chemotherapy regimen + recombinant human endostatin 7.5 0 mg/m^2^, 0.9% sodium chloride injection 500 ml, once a day, *d*_1–14_	21	(1) (2)	2
Jia Xiaoqiong in 2017	20	20	50.00 ± 2.00		Gemcitabine 1.00 mg/m^2^, 0.9% sodium chloride injection 150 ml, intravenous drip, *D*_1_, *D*_8_ + cisplatin 25 mg/m^2^, 0.9% sodium chloride injection 500 ml, intravenous drip, *D*_1–3_	The control group was treated with the chemotherapy regimen + recombinant human endostatin 30 mg, 0.9% sodium chloride injection 110 ml, *D*_1–7_	21	(1) (2) (3) (4) (5)	2
Xu Li in 2017	30	30	54.10 ± 11.30		Gemcitabine 1.00 g/m^2^, 0.9% sodium chloride injection 250 ml, intravenous drip, *D*_1_, *D*_8_ + cisplatin 30 mg/m^2^, 0.9% sodium chloride injection 500 ml, intravenous drip, *D*_1–3_	The control group was treated with the chemotherapy regimen + recombinant human endostatin 15 mg, 0.9% sodium chloride injection 500 ml, intravenous drip, *d*_1–14_	21	(1) (2) (3) (4) (5)	3
Song Wencan in 2018	30	30	61.70	57.40	Gemcitabine 1,250 mg/m^2^, intravenous drip, *D*_1_, *D*_8_ + cisplatin 25 mg/m^2^, intravenous drip, *D*_1–3_	The control group was treated with the chemotherapy regimen + recombinant human endostatin 15 mg/m^2^, intravenous drip, *D*_1–7_	21	(1) (2) (3) (4) (5)	1
Wang Zhifeng in 2018	30	34	55.45	55.97	Gemcitabine 1,000 mg/m^2^, 0.9% sodium chloride injection 100 ml, intravenous drip, *D*_1_, *D*_2_ + cisplatin 75 mg/m^2^, 0.9% sodium chloride injection 500 ml, intravenous drip, divided into 3 days	The control group was treated with the chemotherapy regimen + recombinant human endostatin 15 mg, 0.9% sodium chloride injection 250 ml, intravenously pumped, *d*_1–9_	21	(1) (2) (3) (4) (5)	1
Zhong Li in 2018	25	25	70.34	70.21	Gemcitabine 1,000 mg/m^2^, 150 ml of 0.9% sodium chloride injection, intravenous drip, *D*_1_, *d*_8_ + cisplatin 30 mg/m^2^, 0.9% sodium chloride injection 500 ml, intravenous drip, *D*_1–3_	The control group was treated with the chemotherapy regimen + recombinant human endostatin 7.50 mg/m^2^, 0.9% sodium chloride injection 100 ml, intravenous drip, *d*_1–14_	21	(1) (2) (3) (4) (5)	2

The article "Systematic Evaluation Meta-Analysis of the Efficacy of Recombinant Human Endostatin Combined with Gemcitabine and Cisplatin in Non-Small-Cell Lung Cancer" was published in 2022. Journal: J Healthc Eng.

**Table 2:** Forest map of meta-analysis of patients' efficiency among groups.

Study details	Experimental		Control		Weight (%)	Risk ratio
	Events	Total	Events	Total		MH, fixed, 95% CI
Si Feng, 2012	17	40	9	32	4.1	1.51 [0.78, 2.93]
Fu Hao, 2015	19	32	9	28	3.9	1.85 [1.00, 3.40]
Jian-Wu Liu, 2012	12	30	11	30	4.5	1.09 [0.57, 2.07]
Liu Tao, 2015	21	32	13	32	5.3	1.62 [0.99, 2.63]
Song Wenxian, 2018	16	30	10	30	4.1	1.60 [0.87, 2.94]
Yuan-yuan Zhang, 2014	14	31	9	28	3.8	1.41 [0.72, 2.73]
Xu Li, 2017	11	35	8	35	3.2	1.38 [0.63, 3.00]
Fang Li, 2017	14	23	7	23	2.8	2.00 [0.99, 4.03]
Li Lihua, 2016	13	23	9	23	3.7	1.44 [0.77, 5.69]
LuanWenQiang, 2012	11	25	7	27	2.7	1.70 [0.78, 3.69]
Relapsed Chicken, 2012	67	94	31	90	12.9	1.76 [1.27, 2.44]
Hi-Feng Wang, 2018	19	34	9	30	3.9	1.88 [1.00, 3.47]
Wang Fang, 2011	13	31	11	29	4.6	1.11 [0.59, 2.06]
Mention, 2010	9	20	2	20	0.8	4.50 [1.11, 18.27]
Xie Yanru, 2008	9	22	7	26	2.6	1.52 [0.68, 3.41]
Tany, 2013	21	38	12	38	4.9	1.75 [1.01, 3.03]
Xiao-jing Jia, 2017	6	20	4	20	1.6	1.50 [0.50, 4.52]
Deng Qingping, 2011	5	22	2	18	0.8	2.65 [0.59, 11.88]

Heterogeneity: chi^2^ = 1.75, *d*_*f*_ = 2 (*P* = 0.42), and *I*^2^ = 0%. Test for overall effect: *Z* = 1.23 (*P* = 0.22).

**Table 3:** Forest map of meta-analysis of benefit rate between groups.

Study details	Experimental		Control		Weight (%)	Risk ratio
	Events	Total	Events	Total		MH, fixed, 95% CI
Si Feng, 2012	32	40	18	32	3.5	1.42 [1.01, 2.00]
Fu Hao, 2015	28	32	22	28	4.1	1.11 [0.88, 1.41]
Jian-Wu Liu, 2012	25	30	19	30	3.3	1.32 [0.96, 1.80]
Liu Tao, 2015	31	32	24	32	4.2	1.29 [1.05, 1.59]
Song Wenxian, 2018	25	30	22	30	3.9	1.14 [0.87, 1.49]
Yuan-yuan Zhang, 2014	22	31	19	28	3.5	1.05 [0.74, 1.47]
Xu Li, 2017	30	35	22	35	3.9	1.36 [1.02, 1.82]
Fang Li, 2017	20	23	12	23	2.3	1.54 [1.04, 2.28]
Li Lihua, 2016	23	23	22	23	4.0	1.04 [0.93, 1.18]
LuanWenQiang, 2012	20	25	14	27	2.4	1.54 [1.02, 2.33]
Relapsed Chicken, 2012	87	94	71	90	12.8	1.17 [1.04, 1.32]
Hi-Feng Wang, 2018	28	34	21	30	3.9	1.18 [0.89, 1.56]
Wang Fang, 2011	27	31	22	29	4.0	1.15 [0.90, 1.47]
Mention, 2010	20	20	18	20	3.3	1.11 [0.93, 1.31]
Xie Yanru, 2008	17	22	19	26	3.1	1.06 [0.76, 1.46]
Tany, 2013	34	38	24	38	4.2	1.42 [1.09, 1.85]
Xiao-jing Jia, 2017	16	20	12	20	2.1	1.33 [0.88, 2.03]
Deng Qingping, 2011	11	17	6	18	1.0	1.94 [0.92, 4.08]

Heterogeneity: chi^2^ = 1.75, *d*_*f*_ = 2 (*P* = 0.42), and *I*^2^ = 0%. Test for overall effect: *Z* = 1.23 (*P* = 0.22).

The article "Systematic Evaluation Meta-Analysis of the Efficacy of Recombinant Human Endostatin Combined with Gemcitabine and Cisplatin in Non-Small-Cell Lung Cancer" was published in 2022. Journal: J Healthc Eng.

## Data Availability

The data used to support this study are available from the corresponding author upon request.
